# Research on Diagnostic Information of Smart Medical Care Based on Big Data

**DOI:** 10.1155/2021/9977358

**Published:** 2021-06-02

**Authors:** Zhihai Xu, Donglin Shi, Zhiwei Tu

**Affiliations:** ^1^School of Information Engineering, Nanchang University, Nanchang 330031, Jiangxi, China; ^2^Health Development Center of Jiangxi Province, Nanchang 330006, Jiangxi, China; ^3^Information Office, The First Affiliated Hospital of Nanchang University, Nanchang 330006, Jiangxi, China

## Abstract

The medical field has gradually become intelligent, and information and the research of intelligent medical diagnosis information have received extensive attention in the medical field. In response to this situation, this paper proposes a Hadoop-based medical big data processing system. The system first realized the ETL module based on Sqoop and the transmission function of unstructured data and then realized the distributed storage management function based on HDFS. Finally, a MapReduce algorithm with variable key values is proposed in the data statistical analysis module. Through simulation experiments on the system modules and each algorithm, the results show that because the traditional nondistributed big data acquisition module transmits the same scale of data, it consumes more than 3200 s and the transmission time exceeds 3000 s. The time consumption of smart medical care under the 6G protocol is 150 s, the transmission time is 146 s, and the time is reduced to 1/10 of the original. The research of intelligent medical diagnosis information based on big data has good rationality and feasibility.

## 1. Introduction

With the continuous progress of society and the improvement of human living standards, the guarantee of the quality of human life is closely related to the problems in the medical field. Use cloud computing, Internet of Things, data mining, and other related information technologies to closely link patients with medical staff, medical institutions, and medical equipment to promote comprehensive medical informatization. This model aims to improve service efficiency, implement the service concept of always taking the patient as the center, and truly optimize the services of the medical system. Governments, companies, and researchers have begun to study the application of big data in smart healthcare.

Scholars and researchers at home and abroad have conducted research on the theory and practice of intelligent medicine. These problems not only cause the waste of medical resources and human and financial resources but also make the contradiction between doctors and patients in our country increasingly acute and have a certain negative impact on the harmonious and healthy development of society. Shang Yanan proposed a privacy-protected intelligent medical diagnosis system. In IMDS, users submit health check parameters to the server in a protected form. The server then retrieves the most likely disease from the database and returns it to the user. In the above search process, we used casual keyword search as the basic framework, so that the server could not obtain any personal information from the user's data while maintaining computing power. In addition, this article also provides a method for preprocessing the data stored on the server side to make the protocol more efficient. However, his research did not clearly propose how a privacy-protecting intelligent medical diagnosis system does not disclose information [1]. The HIS proposed by Yang Yiqi is a hierarchical integration of incremental learning fuzzy neural network (ILFN) and a fuzzy language model optimized by genetic algorithm. ILFN is a self-organizing network with fast, online, and incremental learning capabilities. The language model is based on the knowledge embedded in the trained ILFN. The knowledge gained from the low-level ILFN can be mapped to the high-level language model and vice versa. The genetic algorithm is used to optimize the language model to maintain high accuracy and comprehensibility. The resulting HIS can handle low-level numerical calculations and high-level language calculations. After the system is completed, you can gradually learn the new information in the digital structure and language structure. In order to evaluate the performance of the system, the benchmark data of breast cancer was studied as a medical diagnosis application. The simulation results show that the performance of the proposed HIS system is better than that of a single independent system, but its overall research lacks data support, and more data is needed to support its conclusions [2]. Wang Zeyun proposed a new intelligent prediction system that uses feature-selected medical data sets to more accurately predict the occurrence of heart disease. For this reason, a new weighted genetic algorithm is proposed to select very important features from the data set to improve the accuracy of disease prediction. In this intelligent prediction system, a new weighted genetic algorithm is used to preprocess the data, and a new weighted fuzzy C-means clustering algorithm is used for effective segmentation. Finally, we use the ID3 algorithm for classification, which helps to make effective decisions. The experimental results lack more data support so that it is still doubtful whether the prediction accuracy of the disease can be improved [3].

This article coordinates the orderly collaboration of various medical departments to manage medical staff more effectively. The system first realized the ETL module based on Sqoop and the transmission function of unstructured data and then realized the distributed storage management function based on HDFS. Finally, a MapReduce algorithm with variable key values is proposed in the data statistical analysis module. Through the simulation experiment of the collection module and the statistical analysis method of the system, the results show that the design and implementation of the system have certain advantages. Based on this system, an Apriori algorithm based on Boolean matrix operations is also proposed here. Through comparative experiments on the Apriori algorithm before and after the improvement, the results show that the algorithm is simple and fast and can extract various relevant patterns from a large number of electronic medical records, thereby achieving the purpose of auxiliary dispensing.

The chapters of this article are arranged as follows: Section 1 is devoted to introduction and mainly emphasized the research significance of intelligent medical diagnosis information based on big data, the classification of intelligent medical diagnosis systems, and the current status and development trend of research and development in the medical information industry at home and abroad.  Section 2 discusses the construction of big data collection modules and big data storage modules and introduces big data statistical analysis methods and intelligent auxiliary diagnosis methods.  Section 3 mainly introduces the data sources, experimental environment, and important algorithms used in the implementation of the system.  Section 4 discusses the comparison of distributed big data collection system architecture verifying the superiority of the big data collection module proposed in this article.  Section 5 summarizes and emphasizes the promotion of computer technology and information processing technology to the medical industry and further looks forward to the intelligent diagnosis system for human beings, as well as contributions made.

## 2. Proposed Method

### 2.1. Big Data Collection Module

As a traditional IT architecture, relational databases cannot do anything in the face of big data. In contrast, Hadoop is a delight to handle all types of big data processing. Hadoop includes HDFS and MapReduce. The former provides big data storage capability for low-latency, high-throughput access. The latter is Hadoop's computing framework and programming framework [4, 5]. Applications developed using the MapReduce programming framework can get the powerful computing power of the Hadoop cluster to handle storage. However, medical big data stored in file systems or relational databases is not very convenient for Hadoop to access and process. On the other hand, distributed applications based on Hadoop can directly exert data pressure on existing clinical data centers, and frequent data access and analysis will put tremendous pressure on clinical business systems. Therefore, it is the best way to collect the required medical big data and store it on HDFS for analysis and processing [6, 7].

This paper designs and develops a Sqoop-based ETL module for structured data stored in the relational database system. The distributed processing features of this module greatly accelerate the process of medical data transmission and optimize the secondary utilization of medical big data. Regarding prerequisites, when transferring data, the ETL module first establishes a connection with the data source through Java Database Connection (JDBC) and looks at the metadata information of the data source and then converts the SQL type data obtained by the JDBC side into a Sqoop record in the Java class format and formats it as a format [8, 9]. Enter the submission to the MapReduce task. Finally, data is written to HDFS by initiating a corresponding number of Map tasks and Reduce tasks. For semistructured and unstructured data, directly call the HDFS file system API to write to HDFS. At the beginning of the write file, the client node calls the HDFS API, and the entire file is divided into packets, and the data packet is managed in the form of a data queue and is awaiting processing. Then, apply for a new data block to the NameNode and obtain a set of DataNodes to store the data block replicas. The DataNode forms a pipeline, which in turn writes the data packets to the corresponding DataNode. When the last DataNode data is written, the confirmation information is returned in the reverse direction, and, finally, the NameNode is submitted to indicate that the writing is completed [10, 11].

### 2.2. Big Data Storage Module

Distributed storage and management of medical data is a key part of Hadoop's medical big data analytics system and the foundation for smart healthcare. Before the raw medical data is distributed and processed, it is first necessary to install Hive and HBase on the named node and then use the Java API provided by the Sqoop tool to connect with the traditional medical database. Then, for the various types of data that needs to be imported, the structural nature is judged:

1. If it is structured data, the Sqoop tool will connect to Hive through the JDBC/ODBC interface and then query whether the stored form corresponding to the data already exists. If it does not exist, create a new table and store it in Hive; if it already exists, determine whether the data volume exceeds the set threshold. If it does not exceed the set threshold , directly save it to Hive; if it exceeds, you need to add the partition and then store it in Hive [12].
2. When the data is unstructured, the Sqoop tool will connect to HBase through the HBase interface and submit the insert request; after the request is responded to, the HBase table is scanned and the insertion position is located, and the timestamp is set and the data is inserted into the HBase database.

To correctly write data to the HDFS distributed file system, the Hadoop cluster needs to be configured accordingly, including the running parameters of the daemon and the Hadoop running environment. After the Hadoop cluster is configured and the original data is successfully imported, the client starts to create the distributed file system HDFS. The data writing process is as follows:

1. The data layer client development library (Client) starts the data node and initiates an RPC connection access request to the named node of the access control layer.
2. The named node checks whether the file to be created already exists and the creator's operating authority is successful and creates a record for the file; if the check fails, an exception is thrown to the client.
3. After the RPC write request is responded to, the client development library (Client) divides the file to be written into multiple packets and then applies for new blocks to the named node and maps the local file to the HDFS data block. The list generation “block report” is submitted to the named node.
4. The named node returns the configuration information of the managed data node to the client, and the client will write to each data node in the form of a pipe (Pipeline) according to the IP address of the data node [13, 14].

### 2.3. Big Data Statistical Analysis Method

At present, when hospitals conduct medical data statistics, most of them use SQL statements to query medical databases, while single-node databases take a long time in traversing data. As data capacity continues to grow, traditional databases can no longer meet the need of high speed of statistical analysis (Algorithms 1 and 2).

In the actual implementation process, the algorithm first determines whether the received key value is an integer, and the integer represents the age and is classified into the corresponding age group. Then regroup the patient group into a key value and determine whether this key value already exists in the Hash Table. If it does not exist, add it to the Hash Table; if it already exists, it will correspond to the value in the Hash Table. Because the existing programming language is designed to use the two-dimensional array when designing the statistical counting class analysis algorithm, the two-dimensional array cannot meet the processing requirements of the Reduce merging of the key values of different numerical types in the Map/Reduce model [15, 16]. Therefore, the algorithm effectively solves the above problem by creating a hash table and using the hash table to support the characteristics of any key-value pair.

### 2.4. Intelligent Assistant Diagnosis Method

#### 2.4.1. Apriori Association Analysis Algorithm

The Apriori algorithm is one of the most classic algorithms among many associated algorithms, and its main purpose is to find frequent itemsets. It was proposed by Agrawal et al. in 1994.

- Step 1: set the minimum support and confidence according to user requirements
- Step 2: build a candidate 1-item set
- Step 3: construct a candidate 2-item set from the frequent 1-item set through the join step and the pruning step, and generate the frequent 2-item set as in step 2
- Step 4: repeat step 3 until you cannot create a candidate set

Among the above four steps, there are two key operations, connection and pruning, which are described as follows.

In the connection step, first, a set of candidate k-item sets is generated from the (*k* − 1)-item set by connection, denoted as Ck. Let *l*1 and *l*2 be the item set in *Lk* − 1, and Li represents the *j*th item in li. If the first (*k* − 2) terms in *l*1 and *l*2 are the same (sorted by dictionary), then *l*1 and *l*2 are frequent (*k* − 1)-item sets that can be joined, from which candidate k-items are generated; and its form is *L*1 [1], *L*1 [2], ..., *L*1[*k* − 2], *L*1[*k* − 1], *L*2[*k* − 1] [17, 18].

In the pruning step, Ck is a superset of Lk, and its members may not be frequent.

The absolute power is a value used to calculate the absolute value of the brain's electrical power.

(1) $$\begin{array}{c} \text{AP}=10\;\log\;P. \end{array}$$

In the above formula,*P* represents the power value of brain electricity.

(2) $$\begin{array}{c} \text{RP}=10\;\log\frac{P}{\text{Carrier}}. \end{array}$$

For any spectrum *U*(*f*, *t*), there are

(3) $$\begin{array}{c} f_{c,t}=\frac{\int_{-\infty }^{\infty }fU\left(f,t\right)\text{d}f}{\int_{-\infty }^{\infty }U\left(f,t\right)\text{d}f},\\ \sigma_{t}^{2}=\frac{\int_{-\infty }^{\infty }{\left(f-f_{c,t}\right)}^{2}U\left(f,t\right)\text{d}f}{\int_{-\infty }^{\infty }U\left(f,t\right)\text{d}f}. \end{array}$$

The center frequency is used in research related to EEG and memory. The absolute center frequency is used to calculate the value of the absolute center frequency of the EEG signal [19, 20].

(4) $$\begin{array}{c} \text{ACF}=\left|{\text{CF}}_{\alpha }-{\text{CF}}_{b}\right|. \end{array}$$

In the above formula, CF represents the center frequency of *α* point.

#### 2.4.2. Apriori Algorithm Based on Matrix Operation

In this paper, the Apriori algorithm based on matrix operation is adopted. A library of things is represented by a Boolean matrix. When searching the frequency of the item set, scan the column corresponding to the Boolean matrix, and find the frequency of the k-item set {*I*1, *I*2, ..., *Ik*}, only need to be the first, second,... of the matrix, The k-column vector performs a bitwise AND operation and then counts 1 in the result of the vector operation [21, 22]. Repeat steps 2-3 and continue to perform matrix compression. On the one hand, the size of the matrix can be reduced, and, on the other hand, the efficiency of the algorithm can be improved. Then, proceed to step 4 until Lk is empty and the algorithm terminates.

## 3. Experiments

### 3.1. Data Source

To better verify the feasibility and superiority of the method, the experimental data is selected from medical big data collected by large domestic comprehensive hospitals. The electronic medical records of patients were obtained from the electronic HIS system of a top-three hospital in Zhejiang Province, with a total of 128 GB of medical data. The dataset counts information about patients who visited the hospital from January 1, 2014, to January 1, 2018, including 132,097 patients and more than 100 million records.

### 3.2. Experimental Environment

The main hardware devices used in the experiment mainly include medical servers, personal PCs, fiber switches (Switch), and disk array storage platforms. The system is developed using Java language tools. The built Hadoop cluster runs on the Linux operating system platform. The list of experimental software devices is shown in Table 1.

In this experiment, the medical big data processing system is built on a Linux cluster with 5 nodes, a NameNode, and four DataNodes, each with Hadoop distributed architecture software installed. The user interface and the computing center are all encapsulated in the NameNode, and the Hive and HBase databases and the data export tool Sqoop are installed. All user operations will be completed in the NameNode.

## 4. Results and Discussion

The superiority of the big data collection module in this paper is verified by comparing the distributed system architecture with the traditional nondistributed big data collection. The big data collection module speeds up the data transmission by initiating Map and Reduce tasks and needs to find a balance between the cluster performance and the number of tasks in a specific cluster configuration. Therefore, this paper guarantees as much as possible that there is no difference in experimental configuration except for distributed and nondistributed differences. The comparative experimental results of the big data collection module are shown in Figure 1. The adverse reactions during the treatment are shown in Table 2. The results of the adverse reaction analysis are shown in Figure 2.

Figure 1 shows the results of a comparison of big data collection modules in distributed and nondistributed systems. Because the traditional nondistributed big data collection module transmits the same scale data, the consumption time exceeds 3200 s, and the transmission time exceeds 3000 s. The time consumption of smart medical care under the 6G protocol is 150 s, the transmission time is 146 s, and the time is reduced to 1/10 of the original. Besides, experiments have shown that the number of Map and Reduce tasks may slow down the overall transmission time as the cluster performance is saturated. In this paper, the distributed big data collection module can increase the number of DataNodes to increase the threshold of the number of Map and Reduce tasks, thus reducing the time consumption rate and reducing the consumption time. The consumption time of the collection module of the nondistributed system is positively related to the data size; that is, when the data size is larger, the time consumption will increase linearly.

In this paper, through the MapReduce operation of 60532 electronic medical records, the statistical analysis method of this paper is compared with the classical database. The experimental results recorded are shown in Table 3.

The results of the comparison between the statistical analysis method and the classic data SQL server are shown in Figure 3.

Besides, with the increase in the number of processed electronic medical records, the traditional single-node database time consumption has a linear growth trend; and, in the Hadoop-based medical big data analysis system, because of the distributed processing method in the data statistics process, time consumption has not increased significantly. The influence of covariates on the trajectory of quality-of-life changes is shown in Table 4. The impact of disability acceptance on the quality of life of burn patients is shown in Table 5. The analysis of the influence of covariates on the trajectory of quality-of-life changes is shown in Figure 4. The analysis of the impact of disability acceptance on the quality of life of burn patients is shown in Figure 5.

By comparing the performance of the Apriori algorithm before and after the improvement, the superiority is verified. The experimental results are shown in Figure 6. The accuracy of different features in different brain wave frequency bands is shown in Table 6. The treatment effect is shown in Figure 7.

Under the same conditions, the running speed is improved, and the performance of frequent itemset discovery is improved. Therefore, the Apriori algorithm based on the Boolean matrix operation proposed in this paper can dig out various correlation modes from a large number of electronic medical records in a short time, thus achieving the purpose of auxiliary dispensing. The 2DE, 3DE, X-ray images, and the measured values (mm) of the ASD size of the measurement board are shown in Table 7. The comparison of the three methods for ASD size measurement is shown in Figure 8.

## 5. Conclusions

Under the new network protocol, the smart medical system improves the operating speed and improves the performance of frequent itemset discovery. The Apriori algorithm based on Boolean matrix operation can dig out various related patterns from a large number of electronic medical records in a short time to achieve the purpose of assisting glue dispensing.

The continuous improvement of people's living standards has made people pay more and more attention to their health. However, with the aging of China's population, the problem of environmental pollution has become more and more serious. At the same time, due to the increase of modern life and work pressure, the number of patients with various chronic diseases has also increased. Through the smart medical platform and sensory terminal, Smart Medical can realize the health diagnosis, intelligent diagnosis of diseases, and follow-up treatment and management of diseases, which can realize remote detection and analysis, diagnosis, and treatment, so that users can know the disease situation in time and the early stage of the disease and get timely detection and treatment. In recent years, the Chinese government, scientific research institutions, and major companies have paid great attention to the development of the smart medical field and vigorously promoted the advancement of smart medical care.

At present, China's research in the field of smart medical care is in its infancy. The existing smart medical systems generally have problems such as high system erection cost, poor data storage reliability, and weak data processing capability. The system implements the transmission function of the ETL module and unstructured data based on Sqoop and then implements the function of distributed storage management based on HDFS. Finally, the MapReduce algorithm with variable key value is proposed. Through the simulation experiments on the system module and each algorithm, the results show that the research on the diagnostic information has good rationality and feasibility.

## Figures and Tables

**Figure 1:** Comparison of experimental results of the big data collection module.

**Figure 2:** Adverse reaction analysis results.

**Figure 3:** Comparison of experimental results of big data analysis methods.

**Figure 4:** Analysis of the influence of covariates on the trajectory of quality of life.

**Figure 5:** Analysis of the impact of disability acceptance on the quality of life of burn patients.

**Figure 6:** Comparison of experimental results of Apriori algorithm before and after improvement.

**Figure 7:** Treatment effect.

**Figure 8:** Comparison of ASD size measurement by three methods.

**Algorithm 1:** The implementation process of the Mapper algorithm.

**Algorithm 2:** The Reducer algorithm.

**Table 1:** List of experimental software devices.

Device name	Version number
Development tools	JDK 1.7
Operating system	Ubuntu Linux 14
Distributed cluster	Hadoop 2.6.28

**Table 2:** Adverse reactions during treatment.

Symptom	Group		
	Observation group (*n* = 55)	Control group (*n* = 53)	*P*
Dizziness	2 (3.6)	1 (1.8)	0.36
Insomnia	1 (1.8)	0	0.51
Nausea	1 (1.8)	0	0.51
Neck	1 (1.8)	0	0.51
Pain	0	1 (1.8)	0.51
Headache	0	1 (1.8)	0.51
Inattention	0	1 (1.8)	0.51

**Table 3:** Comparison table of big data analysis methods.

Number of electronic medical records	Big data statistical analysis method	Traditional database
10000	105	2187
20000	152	4127
30000	164	6401
40000	190	8785
50000	201	11023
60000	252	13242

**Table 4:** The influence of covariates on the trajectory of quality of life.

Value		Parameter		
		Estimated value	*T*	*P*
Gender	Intercept	−0.121	−0.045	0.964
	Slope	−0019	0.073	D.942

Causes of burns	Intercept	−0.469	0.580	0.562
	Slope	−0.067	0.854	0.393

Severity	Intercept	−10.721	−6.229	<0.001
	Slope	0.126	0.719	0.472

Complications	Intercept	5.522	1 977	0.048
	Slope	0.508	1 857	0.063

Payment methods	Intercept	0.117	0.136	0 892
	Slope	−0.041	−0.498	0.619

Education level	Intercept	0.35	0.314	0.754
	Slope	−0.118	−1.078	0.281

**Table 5:** The impact of disability acceptance on the quality of life of burn patients.

Time		Parameter		
		Regression coefficient	*T*	*P*
ADS (at discharge)	BSHS (upon discharge)	0.616	18.874	<0.001
ADS (1 month after hospital)	BSHS (1 month after hospital)	0.669	21. 660	<0.001
ADS (3 months after hospital)	BSHS (3 months after hospital)	0.681	22. 824	<0.001
ADS (6 months after hospital)	BSHS (6 months after hospital)	0.678	22..123	<0.001

**Table 6:** Accuracy of different features in different brain wave frequency bands.

Feature	Brain waves					
	Delta (%)	Theta (%)	Alpha (%)	Beta (%)	Gamma (%)	All (%)
Devolatility	59. 57	66.13	68.39	80.23	81.97	86 87
Hurst index	43.1 9	45.4 6	53. 1 0	62.74	66.79	75.06
Squared difference	61.76	64. 69	67.78	69.76	70.79	80.09
Approximate entropy	72. 89	73. 68	75. 38	74.1 2	73.8 2	82.65

**Table 7:** ASD size of 2DE, 3DE, X-ray images, and measured values of the measuring board (mm).

Measurement methods	Measured value	*P*	*r*
X-ray image measurement	23.59 ± 8.82	<0.001	0.97
Two-dimensional ultrasonic measurement (upper and lower diameter)	19.65 ± 7.60	<0.001	0.97
Three-dimensional ultrasonic measurement (upper and lower diameter)	20. 82 ± 7.43	<0.001	0.92
Two-dimensional ultrasound + balloon measurement	24.17 ± 7.94	>0.05	0.97

## Data Availability

No data were used to support this study.
